RETRACTED

# Comparative Evaluation of the Incidence of Postoperative Pulmonary Complications After Minimally Invasive Valve Surgery vs. Full Sternotomy: A Systematic Review and Meta-Analysis of Randomized Controlled Trials and Propensity Score-Matched Studies

**DOI:** 10.3389/fcvm.2021.724178

**Published:** 2021-08-23

**Authors:** Mohamed Abdulkadir Mohamed, Shuai Ding, Sayed Zulfiqar Ali Shah, Rui Li, Najib Isse Dirie, Cai Cheng, Xiang Wei

**Affiliations:** ^1^Division of Cardiothoracic and Vascular Surgery, Tongji Hospital, Tongji Medical College, Huazhong University of Science and Technology, Wuhan, China; ^2^Department of Rehabilitation Medicine, Tongji Hospital, Tongji Medical College, Huazhong University of Science and Technology, Wuhan, China; ^3^Division of Urology, Tongji Hospital, Tongji Medical College, Huazhong University of Science and Technology, Wuhan, China

**Keywords:** cardiac surgery, minimally invasive, valve repair/replacement, meta-analysis (as topic), full sternotomy

## Abstract

**Background:** Postoperative pulmonary complications remain a leading cause of increased morbidity, mortality, longer hospital stays, and increased costs after cardiac surgery; therefore, our study aims to analyze whether minimally invasive valve surgery (MIVS) for both aortic and mitral valves can improve pulmonary function and reduce the incidence of postoperative pulmonary complications when compared with the full median sternotomy (FS) approach.

**Methods:** A comprehensive systematic literature research was performed for studies comparing MIVS and FS up to February 2021. Randomized controlled trials (RCTs) and propensity score-matching (PSM) studies comparing early respiratory function and pulmonary complications after MIVS and FS were extracted and analyzed. Secondary outcomes included intra- and postoperative outcomes.

**Results:** A total of 10,194 patients from 30 studies (6 RCTs and 24 PSM studies) were analyzed. Early mortality differed significantly between the groups (MIVS 1.2 vs. FS 1.9%; *p* = 0.005). Compared with FS, MIVS significantly lowered the incidence of postoperative pulmonary complications (odds ratio 0.79, 95% confidence interval [0.67, 0.93]; *p* = 0.004) and improved early postoperative respiratory function status (mean difference −24.83 [−29.90, −19.76]; *p* < 0.00001). Blood transfusion amount was significantly lower after MIVS (*p* < 0.02), whereas cardiopulmonary bypass time and aortic cross-clamp time were significantly longer after MIVS (*p* < 0.00001).

**Conclusions:** Our study showed that minimally invasive valve surgery decreases the incidence of postoperative pulmonary complications and improves postoperative respiratory function status.

RETRACTED

## Introduction

Full median sternotomy (FS) has long been the standard incision for cardiac surgery due to it is excellent exposure of the heart and great vessels. However, to reduce the size of the sternotomy, cardiac surgeons have long pursued less extensive incisions to improve outcomes and thus have used minimally invasive approaches that have undergone rapid development in the last few decades (1–3). These approaches have multiple benefits over an FS because of a smaller surgical incision, reduced pain, earlier discharge, and quicker postoperative recovery (4, 5). On the other hand, some potential technical disadvantages tend to have prolonged cardiopulmonary bypass (CPB) and aortic cross-clamp time (6, 7).

Given such developments in surgical management and patients' treatment over the years, postoperative pulmonary complications remain a leading cause of mortality and morbidity following cardiac surgery (8, 9). These complications contribute to longer hospital stays and more readmissions into the ICU, significantly affecting health care and increasing healthcare systems' financial burden (8, 10). Atelectasis and pleural effusions, pneumonia, pneumothorax, diaphragm paralysis because of phrenic nerve damage, and pulmonary infection are the most common pulmonary complications (11).

Although considerable benefits were associated with the MIVS over FS, there is still ongoing debate about the advantage of MIVS on postoperative pulmonary complications (PPCs), and the associations remain unclear. To our knowledge, there is still limited evidence on PPCs and respiratory system function analysis of patients after MIVS compared with the FS approach has not been analyzed. Therefore, based on the existing clinical literature, we conducted this systematic review and meta-analysis of high-quality randomized controlled trials (RCTs) and propensity score-matched (PSM) studies to analyze the incidence of PPCs and respiratory function of patients who underwent a minimally invasive approach for mitral or aortic valve vs. FS.

## Methods

### Selection Criteria

We included all articles reporting clinical outcomes for MIVS (repair or replacement of the mitral valve, aortic valve, or both valves) via right/lateral mini-thoracotomy or mini-sternotomy, with either a camera or direct visualization, vs. traditional FS. Studies were considered using a PICOS (Population, Intervention, Comparison, Outcome, and Study) strategy if (1) articles were published in English, (2) articles reported RCTs or PSM studies, (3) articles compared the outcomes of MIVS and FS for either mitral or aortic valve disease, and (4) outcomes included postoperative pulmonary complications and early postoperative respiratory function.

RETRACTED

Articles without a full report available, review studies, studies with previous cardiac surgery and concomitant surgical procedures (coronary artery bypass grafting, and procedure involving ascending aortic) other than isolated mitral and aortic or both valve surgery were excluded and studies with no comparison group were also excluded.

### Information Sources

The following databases were used: PubMed, MEDLINE, Web of Science, Cochrane Central Register of Controlled Trials, Scopus, and Google Scholar. The reference lists of identified articles were also included in manual searches.

### Search Strategy

We searched articles and studies comparing FS vs. MIVS using the following medical subject headings: aortic valve, aortic valve surgery, mitral valve or mitral valve surgery, minimally/partial invasive, full/conventional/partial sternotomy or mini-sternotomy, anterolateral/right mini-thoracotomy, partial upper Hemi-sternotomy or upper mini-sternotomy.

### Study Selection

Search strategies, inclusion with exclusion criteria, statistical analysis, and outcomes were predefined. Thirty publications fulfilled our eligibility criteria (5, 6, 12–39). Two independent investigators (MA, SZ) reviewed all abstracts that fulfilled the search criteria. When there were differences of opinion between these investigators, other authors were included to resolve disagreements. Figure 1 summarizes the search strategy.

**Figure 1:** Flowchart for studies included in data search in accordance with PRISMA guidelines.

### Data Extraction

Two reviewers independently extracted data from each included study and performed the quality assessment. Data extracted included the first author's name, year of publication, country, study interval, study type, the number of subjects who underwent MIVS or FS, and outcomes of interest. The following clinical outcomes of interest from each study were extracted to compare MIVS with FS: postoperative pulmonary complications (overall complications, pneumonia, pleural effusion, pneumothorax, pulmonary infection, and respiratory insufficiency), early postoperative pulmonary function variables after 1 week (forced expiratory volume in 1 second [FEV1], forced total lung capacity (TLC), and forced vital capacity [FVC%]). Secondary outcomes of interest included early mortality, blood transfusion and, cardiopulmonary bypass (CPB) time, aortic cross-clamp time, and operative time.

### Risk-of-Bias and Study Quality Assessment

Two independent reviewers (SZAS and NID) assessed the risk-of-bias using the Cochrane risk-of-bias (RoB2) tool. The risk-of-bias was categorized as low, high, or unclear risk-of-bias. The RoB2 Excel tool was applied to individual studies, and results were entered into Cochrane's Review Manager 5.3 (40). The Newcastle–Ottawa Scale (NOS) was used to assess the methodological quality of all observational studies. The NOS assesses the following characteristics of a study: selection of the general population, comparability, and adequate assessment of outcomes, to evaluate the methodological quality of studies (41). Based on the NOS, a maximum of 9 points can be given to each study. In this review, the modified NOS scores ≥ 7 were considered to indicate high-quality publications. Furthermore, the methodological quality of RCTs was assessed using the Jadad scale, which evaluates RCT quality using a maximum score of 5. A Jadad score ≥ 3 was considered to indicate high-quality RCTs (42).

RETRACTED

### Definitions of Outcomes

MIVS was defined as any procedure not performed with an FS. A full sternotomy was performed from the sternal notch to the xiphoid process. The definitions of the postoperative outcomes mainly depend on the descriptions mentioned in the original articles (8, 18, 39, 43–45). Besides postoperative pulmonary complications were defined as complications occurring in the postoperative period and producing clinical diseases, such as pneumonia, pleural effusion, pneumothorax, pulmonary infection, and respiratory insufficiency (defined as the need for reintubation or tracheostomy after initial extubation), and prolonged ventilation time, which was defined as mechanical ventilatory support requirement for more than 24 h. Pulmonary function tests, represented by FEV1, TLC, and FVC, were assessed based on a spirometry test 1 week after surgery. The incidence of early mortality was defined as death in the hospital or within 30 days post-surgery.

### Statistical Analysis

As per Cochrane Collaboration guidelines, all statistical meta-analyses were performed using Review Manager 5.3 software (Cochrane Collaboration, Copenhagen, Denmark). We calculated pooled odds ratios (ORs) with their 95% confidence intervals (CIs) for dichotomous data, which are presented as numbers and percentages. Weighted mean differences (WMDs) were used to assess continuous data, which are presented as means ± standard deviation or medians with interquartile ranges. We assessed the heterogeneity of studies by means of *I*^2^ and chi-square test. As a sensitivity analysis, FS and MIVS from RCTs and from PSM studies were compared separately. The reported results all are two-sided, and a *p* < 0.05 was considered to indicate statistical significance.

## Results

### Characteristics of Eligible Studies

Our literature search revealed 30 studies that met our selection criteria (5, 6, 12–39). The total number of patients in these studies was 10,194; 5,097 (50%) patients underwent MIVS, and 5,097 (50%) patients underwent FS. Six studies were RCTs (*n* = 418 patients) (5, 6, 14–16, 28) and 24 were PSM studies (*n* = 9,776 patients) (12, 13, 17–27, 29–39). The characteristics of these studies are shown in Table 1. Figure 1 shows the PRISMA flowchart of the search and selection strategy (46).

RETRACTED

**Table 1:** Characteristics of included studies.

**References**	**Country**	**Study interval**	**Study type**	**No. of patients MIVS/FS**	**Surgical approach**	**Quality assessment**	**LOE** ^**†**^	**Median follow-up**
Aris et al. (6)	Spain	NS	RCT	20/20	A φ	3/5	2b	6 days
Machler et al. (28)	Austria	1996–1997	RCT	30/30	A φ	3/5	2b	294 days^M^
Bonacchi et al. (14)	Italy	1999–2001	RCT	40/40	A φ	4/5	1b	9.7 ± 5.7 months^M^
Dogan et al. (16)	Germany	2003–2004	RCT	20/20	M §	2/5	3b	NS
Moustafa et al. (5)	Egypt	NS	RCT	30/30	A φ	2/5	3b	NS
Calderon et al. (15)	France	2003–2007	RCT	39/39	A φ	5/5	2b	NS
Albacker et al. (12)	US	1995–2010	PSM	223/223	A §	7	4	2 years
Masiello et al. (29)	Italy	1997–1999	PSM	100/100	A φ	6	3b	1 month
Farhat et al. (17)	France	2000–2001	PSM	50/50	A φ	7	3b	1 month
Tabata et al. (37)	US	1996–2005	PSM	41/41	A φ	7	3b	NS
Iribarne et al. (25)	US	2000–2008	PSM	382/382	M §	8	3b	4.2 ± 2.4 yrs^M^
Holzhey et al. (24)	Germany	1999–2009	PSM	143/143	M §	8	1b	2.4 ± 2.1 yrs^M^
Bang et al. (13)	Korea	1997–2010	PSM	73/73	A ϕ	7	3b	NS
Murzi et al. (31)	Italy	2006–2010	PSM	100/100	A θ	6	2b	3 years
Sansone et al. (32)	Italy	2008–2010	PSM	50/50	A θ	7	3b	NS
Johnston et al. (26)	US	1995–2004	PSM	832/832	A φ	8	3a	6.5 ± 3.0 years^M^
Gilmanov et al. (20)	Italy	2004–2011	PSM	182/182	A θ	7	3b	Until patient discharge
Hiraoka et al. (23)	Japan	2007–2012	PSM	36/36	A ϕ	7	4	NS
Ghanta et al. (19)	US	2011–2013	PSM	289/289	A ϕ	6	4	NS
Gilmanov et al. (21)	Italy	2001–2013	PSM	100/100	A θ	8	3a	33.7 months^M^
Merk et al. (30)	Germany	2003–2012	PSM	477/477	A φ	6	3a	3.1 ± 2.7 years^M^
Shehada et al. (34)	Germany	2002–2012	PSM	585/585	A φ	7	3b	NS
Stoliński et al. (36)	Canada	2010–2013	PSM	211/211	A θ	8	3b	NS
Gasparovic et al. (18)	Slovakia	2010–2013	PSM	34/34	A φ	7	3a	5 years
Levack et al. (27)	US	1995–2014	PSM	483/483	A φ	8	3b	NS
Stolinski et al. (35)	Poland	2011–2014	PSM	212/212	A θ	8	3a	3 months
Seitz et al. (33)	Australia	2013–2016	PSM	53/53	A θ	7	3b	NS
Hawkins et al. (22)	US	2011–2016	PSM	74/74	M §	7	3b	NS
Wang et al. (38)	China	2012–2015	PSM	67/67	M §	6	3a	2.8 years
Zhao et al. (39)	China	2013–2016	PSM	91/91	C δ	8	3a	1 year

*A, Aortic valve; C, indicated both mitral and aorta valve; FS, full sternotomy; LOE, level of evidence; MIVS, minimally invasive valve surgery; M, mitral valve; ^M^, mean; NS, not specified; PSM, propensity score-matching; RCT, randomized control trial; θ, indicates aortic valve surgery right mini-thoracotomy; φ, indicates aortic valve surgery upper mini-sternotomy; ϕ, indicated aortic valve surgery right mini-thoracotomy and upper mini-sternotomy; δ, indicated both mitral and aorta valve surgery right mini-thoracotomy; §, indicated mitral valve surgery right mini-thoracotomy*;

† *Based on US Preventive Services Task Force grading system*.

RETRACTED

The RCTs scored at least 3 out of 5 on the Jadad scale, and most of the PSM studies scored at least 7 out of 9, based on a modified version of the NOS scale (Table 1 and Figure 2). Therefore, overall, the studies were considered to be of high quality.

**Figure 2:** Risk of bias assessment summary.

### Postoperative Pulmonary Complications Outcomes

We analyzed data on postoperative pulmonary complications from 27 studies (6, 12–14, 16–34, 36–39). The overall complications were less in MIVS patients than in FS patients (OR 0.79; 95% CI [0.67, 0.93]; *p* = 0.004). The results of our meta-analysis are summarized in Table 2, and forest plots are shown in Figure 3.

**Table 2:** Overall and subgroup analysis of postoperative respiratory function and complications comparing MIVS and FS.

**Outcome of interest**	**n/N**	**No. patients MIVS/FS**	**Overall effect**	***P***	**Study heterogeneity**			
			**WMD/OR (95% CI)** ^**†**^		**chi^**2**^-test**	**df**	***I*^**2 (%)**^**	***P*-value**
**Postoperative respiratory function status after 1 week**								
**Overall spirometry**	6 (1,928)	964/964	MD −24.83 [−29.90,-19.76]^†^	<0.00001	11770.40	13	100	<0.00001
**Subgroup analysis**								
FEV1%	6 (722)	361/361	−74.06 [−89.14, −58.99]^†^	<0.00001	1089.82	5	100	<0.00001
FVC%	5 (642)	321/321	4.99 [1.23, 8.75]^†^	0.009	287.63	4	99	<0.00001
TLC	3 (564)	282/2,282	8.39 [2.00, 14.78]^†^	0.01	72.03	2	97	<0.00001
**Overall PPCs**	30 (10,194)	5,097/5,097	0.79 [0.67, 0.93]	0.004	28.51	27	5	0.39
RCT	6 (418)	209/209	OR 0.32 [0.12, 0.90]	0.03	4.29	4	7	0.37
PSM	24 (9,776)	4,888/4,888	OR 0.80 [0.69, 0.94]	0.005	20.98	22	0	0.52
**Subgroup analysis**								
Pneumonia	5 (916)	458/458	1.42 [0.44, 4.55]	0.56	2.81	4	0	0.59
Pleural Effusion	8 (1,454)	727/727	0.81 [0.45, 1.45]	0.47	10.28	7	32	0.17
Pneumothorax	4 (420)	210/210	1.55 [0.30, 8.12]	0.60	4.50	3	33	0.21
Respiratory insufficient	12 (5,848)	2,924/2,924	0.75 [0.62, 0.91]	0.004	9.30	11	0	0.59
Pulmonary infection	2 (246)	123/123	1.35 [0.16, 11.30]	0.78	1.24	1	19	0.27
Prolonged ventilation time	10 (3,564)	1,782/1,782	0.72 [0.51, 1.01]	0.06	6.92	9	0	0.65

*n, number of studies; N, number of participants; MIVS, minimally invasive valve surgery; FS, full sternotomy; PPC, postoperative pulmonary complications; WMD, weighted mean difference; OR, odds ratio; CI, confidence interval; I^2^, test of heterogeneity; FEV1, forced expiratory volume in 1 s; FVC, Forced vital capacity; TLC, total lung capacity*;

† *Values of WMD*.

RETRACTED

**Figure 3:** Forest plot demonstrating the overall study incidence of postoperative pulmonary complications between MIVS and FS.

In subgroup analysis, postoperative pulmonary complications differed significantly between the two groups (*p* = 0.0007) in terms of the incidence of postoperative respiratory insufficiency, reported by 12 studies (12, 14, 19, 21, 23, 24, 26, 30, 33, 34, 38, 39) (OR 0.75; 95% CI [0.62, 0.91]; *p* = 0.004). Two studies reported on pulmonary infection: MIVS was associated with a lower chance of infection, but this difference was not significant (OR 1.35; 95% CI [0.16, 11.30]; *p* = 0.78) (13, 17). The incidence of postoperative pleural effusion was reported in 8 studies; this was not significantly different between the groups (OR 0.81; 95% CI [0.45, 1.45]; *p* = 0.47) (6, 16, 18, 20, 21, 28, 29, 36). We also compared the incidence of prolonged ventilation time based on data pooled from 10 studies; there was no significant difference between the groups (OR 0.72; 95% CI [0.51, 1.01]; *p* = 0.06) (14, 19–22, 25, 27, 31, 37, 39). Although the observed proportions of patients with pneumonia (OR 1.42; 95% CI [0.44, 4.55]; *p* = 0.56) and pneumothorax (OR 1.55 95% CI; [0.30, 8.12]; *p* = 0.60) were less among MIVS patients, these were not significantly different between the groups. Subgroup analysis are summarized in Table 2 and forest plots are shown in Figure 4.

**Figure 4:** Forest plot demonstrating the subgroup study of the incidence of postoperative pulmonary between MIVS and FS.

Six studies (5, 6, 14–16, 35) reported on postoperative respiratory function tests based on spirometry, revealing that the overall complications were significantly reduced with MIVS compared to FS (964 vs. 964, WMD −24.83 95% CI [−29.90, −19.76]; *p* = <0.00001). Most pulmonary function tests showed that the MIVS group had better respiratory function than the FS group 1 week after surgery. There was significant heterogeneity among the studies (*p* < 0.00001).

A subgroup analysis of postoperative respiratory function identified that FEV1% (WMD: −78.06; 95% CI [−89.14, −58.99]; *p* < 0.00001), FVC% (WMD: 4.99; 95% CI [1.23, 8.75]; *p* = 0.009), and TLC (WMD: 8.39; 95% CI [2.00, 14.78]; *p* = 0.01) were all significantly better in the MIVS group. There was significant heterogeneity among the studies overall, as well as in the RCT and PSM subgroup (*p* < 0.00001) (Table 2 and Figure 5).

RETRACTED

**Figure 5:** Forest plot demonstrating the incidence of postoperative respiratory function between the MIVS and FS.

### Early Mortality Outcomes

Early mortality was reported as an outcome in 30 studies (5, 6, 12–39), including 5 RCTs (6, 14–16, 28) and 25 PSM studies (12, 13, 17–27, 29–39). The incidence of early death was 1.2 and 1.9% with MIVS, and FS approaches, respectively. Thus, the early mortality rate after MIVS was significantly lower than that after FS (OR 1.58 95% CI: 1.15, 2.16; *p* = 0.005). There was no significant heterogeneity between the groups (*p* = 0.97) (Figures 6A,B).

**Figure 6:** **(A)** Forest plot MIVS vs. FS (Overall early mortality) and **(B)** Funnel plot MIVS vs. FS (overall early mortality).

### Intraoperative Variable Outcomes

MIVS was associated with a significantly prolonged CPB time (WMD: 11.06; 95% CI: 4.29, 17.84 min; *p* = 0.001) (Figure 7) and aortic cross-clamping time (WMD: 23.28; 95% CI: 5.65, 40.87 min; *p* = 0.009) (Figure 8). Thus, the MIVS approach took longer than the FS surgery, although there was no significant difference in the operative time (WMD: 0.39; 95% CI: −0.39, 1.77 h; *p* = 0.32) between the groups (Figure 9). However, the overall heterogeneity between the two approaches was significantly different (*p* < 0.00001). Table 3 provides a summary of these studies.

**Figure 7:** Forest plot of cardiopulmonary bypass time (minutes) between MIVS vs. FS.

**Figure 8:** The forests plot demonstrates aortic cross-clamp time (minutes) between MIVS and FS.

**Figure 9:** The forests plot demonstrates operative time (hours) between MIVS and FS.

**Table 3:** Overall analysis of demographic, intraoperative, and postoperative outcomes comparing MIVS and FS.

**Variables**	**n(N)**	**No. patients MIVS/FS**	**Overall effect WMD/OR (95% CI)** ^**†**^	***P***	**Study heterogeneity**			
					**chi^**2**^-test**	**df**	***I*^**2(%)**^**	***p***
Age, y ± SD	30 (10,194)	5,097/5,097	−0.43 [−1.05, −0.18]^†^	0.17	91.87	29	68	<0.00001
Male, %	27 (9,628)	4,814/4,814	1.01 [0.95, 1.12]	0.48	9.61	26	0	1.00
LVEF %, ± SD	23 (2,910)	3,455/3,455	0.65 [−0.09, 1.39]^†^	0.09	1288.37	22	98	<0.00001
COPD, %	17 (8,132)	4,066/4,066	0.87 [0.74, 1.03]	0.11	4.51	15	0	1.00
Early mortality, %	30 (10,194)	5,097/5,097	0.68 [0.49, 0.95]	0.02	14.42	26	0	0.97
Blood transfusion (unit) ± SD	10 (1,536)	768/768	−0.59 [−2.08, 0.90]^†^	0.44	166.69	9	95	<0.00001
Blood transfusion (patient), %	14 (5,756)	2,878/2,878	0.69 [0.51, 0.93]	0.02	48.53	13	73	<0.00001
CBP time ± SD	27 (8,798)	4,399/4,399	11.06 [4.29, 17.84]^†^	0.001	1924.40	26	99	<0.00001
Cross clamping time, minutes ± SD	28 (9,170)	4,585/4,585	23.28 [5.69, 40.87]^†^	0.009	35361.85	27	100	<0.00001
Operative time, minutes ± SD	13 (2980)	1,490/1,490	0.39 [−0.39, 1.17]^†^	0.32	153.09	12	92	<0.00001

*COPD, chronic obstructive pulmonary disease; CBP, cardiopulmonary bypass; CI, confidence interval; FS, Full sternotomy; I^2^, test of heterogeneity; LVEF, left ventricular ejection fraction; MIVS, minimally invasive valve surgery; n, number of studies; N, number of participants; OR, odds ratio; SD, standard deviation; WMD, weighted mean difference*;

† *Values of WMD*.

RETRACTED

### Need for Blood Transfusion Outcomes

Fourteen studies [2 RCTs (15, 16) and 12 PSM studies (19, 20, 22, 23, 26, 27, 30, 32, 33, 36, 37, 39)] reported on the need for blood transfusion in patients. Twenty-two percent of patients required red blood cell (RBC) transfusion after MIVS, compared to 28% after FS (OR 0.69, 95% CI 0.51, 0.93; *p* = 0.02) (Figure 10).

**Figure 10:** Forest plot of patients transfused red blood cells between MIVS and FS.

Ten studies [3 RCTs (5, 13, 14) and 7 PSM studies (16–18, 24, 31, 36, 38)] reported the units of RBC transfused after MIVS and FS. Those who underwent MIVS used significantly fewer units of RBCs for transfusion than those who underwent FS (WMD −0.59, 95%CI [−2.08, 0.90 U]; *p* = 0.44). There was significant heterogeneity among the studies overall as well for the RCTs and PSM studies (*p* < 0.00001) (Figure 11).

**Figure 11:** Forest plot of units of red blood transfused between MIVS and FS.

## Discussion

Over the past decades, a steady evolution has taken place in the practice of MIVS, with excellent postoperative outcomes, according to the literature. The minimally invasive approach used for the aorta or mitral valve has advantages over the FS method in terms of decreased surgical trauma, postoperative blood loss, and length of ICU and hospital stay (4, 47). Nevertheless, postoperative pulmonary complications remain a common cause of postcardiac surgical morbidity, poor outcomes, increased cost, and hospital stays (48). Therefore, in the context of postoperative pulmonary complications and recovery of early respiratory system function, we considered it necessary to compare MIVS with FS.

In this meta-analysis, we analyzed data of 10,194 patients (5,097 [50%] vs. 5,097 [50%] patients in MIVS vs. FS groups, respectively), from 30 studies (6 RCTs and 24 PSM studies) to evaluate postoperative pulmonary functions status and pulmonary complications after MIVS vs. FS. We also assessed early mortality, CPB time, aortic cross-clamp time, procedure time, and need for blood transfusion between the MIVS and FS. Using the best available level of evidence based on RCTs and PSM studies, our meta-analysis added to the literature that the MIVS is safe and had a significantly reduced overall incidence of postoperative pulmonary complications and respiratory insufficiency and decreased mechanical ventilation time compared with FS.

RETRACTED

Moreover, the overall findings for the secondary outcomes suggested that MIVS, both aortic and mitral, significantly reduced early mortality and blood transfusion requirements. To the best of our knowledge, no previous meta-analyses have indicated whether the incidence of pulmonary complications is lower after MIVS compared with FS. Most studies that describe the effect of cardiac surgery on pulmonary complications were related to patients who underwent a coronary bypass operation through full median sternotomy (49).

It has been reported that the MIVS showed better preserved early postoperative respiratory function status and reduced the time needed to make a full recovery of pulmonary status compared with FS (50). However, there has not been explained this improved respiratory function in the MIVS group so far. This study found that patients undergoing MIVS had a reduced incidence of postoperative pulmonary complications and better postoperative respiratory function outcomes than patients undergoing valve surgery via full median sternotomy. Therefore, we believe that our finding of a reduced incidence of pulmonary complications after the MIVS group may explain the improved lung function than patients with a full median sternotomy. As a result, we believe these phenomena are more likely caused by preserving the chest wall's integrity and reduced surgical trauma. Because of their improved respiratory condition, patients could begin mobilization quicker and perform pulmonary bronchial tree ventilation and cleaning more adequately.

Several risk factors may influence the impairment of spirometry and change in pulmonary gas exchange after cardiac surgery performed via a sternotomy; these include surgical trauma, prolonged operative and CPB time (6, 12, 14, 51). CPB causes an inflammatory cascade of compounds associated with the systemic inflammatory syndrome due to blood interaction with the CPB circuit and decreased pulmonary regeneration, mostly because of insufficient surfactant release triggered by poor perfusion of the alveolar epithelium during CPB (49). Because of the more technical problem, patients in the MIVS group had a longer mean CPB duration than those in the FS group. However, we believe that this variation has no influence impact on postoperative pulmonary complications.

However, if CPB duration were the underlying cause, we would predict the MIVS group to have more significant postoperative pulmonary complications. This study found that patients who underwent MIVS had significantly longer cardiopulmonary bypass time, which may have contributed to the lower number of pulmonary complications observed in this group. A randomized clinical trial would be the only approach to analyze the influence of these independent factors on the incidence of postoperative pulmonary problems. MIVS did not result in an adverse postoperative pulmonary complication. It is likely that patients in whom the MIVS approach was used tended to have better early recovery and more favorable improvement of postoperative pulmonary function because of the shorter mechanical ventilation time, preservation of the chest wall integrity, and reduced postoperative pain, as compared with FS (50, 52, 53). Previous studies drew a similar conclusion to ours: there is less impaired respiratory function among patients who underwent surgery using the MIVS approach (11).

RETRACTED

However, other investigators found no significant differences between the MIVS and FS regarding postoperative respiratory function system improvement (14, 15, 36, 54).

Moreover, we found that patients who underwent MIVS had a significant reduction in the incidence of early mortality (1.2%) compared with FS (1.9%). This finding was in line with that of previously published studies. A study by Mark et al. (30), who analyzed 477 PSM patients who underwent MIVS or FS, showed that MIVS was associated with lower hospital mortality (0.4 vs. 2.3%, respectively). This result was also in line with the results of Paparella et al. (55), who reported on 5,801 patients from different centers who underwent mini-aortic valve replacement vs. conventional aortic valve replacement.

Shehada et al. and Johnston et al. (26, 34) reported on 2,103 and 2,689 patients, respectively, in PSM analyses that compared minimally invasive to conventional aortic valve surgery. They reported a significantly lower incidence of the need for blood transfusion, as well as respiratory insufficiency in MIVS patients. Similarly, we found that the number of patients who required blood transfusion and the number of units of RBC required for transfusion were significantly reduced in MIVS than in FS.

Our observations provide evidence for the value of MIVS as an acceptable alternative option to traditional FS for patients at higher risk of developing pulmonary complications and for patients with chronic lung disease and chronic obstructive pulmonary disease undergoing mitral or/and aortic valve operations (12, 56).

Nevertheless, our study has certain limitations. Most studies did not report similar outcomes, and there was limited information about the pulmonary effects of MIVS. Follow-up for most studies was limited; hence, we were unable to compare long-term results.

RETRACTED

## Conclusions

Based on the above findings in our meta-analysis, MIVS, both mitral and aortic, seem to provide better clinical and surgical outcomes than FS, particularly the benefits of early recovery of postoperative respiratory system functions and reduced incidence of postoperative pulmonary complications. Moreover, MIVS was not associated with an increased incidence of early mortality or a greater need for blood transfusion than FS. We believe that our findings might help surgeons in patient selection, particularly when dealing with patients with a high risk of pulmonary disease undergoing cardiac valve surgical repair or replacement. Finally, further studies comparing MIVS and FS are recommended to validate our findings.

## Data Availability Statement

The raw data supporting the conclusions of this article will be made available by the authors, without undue reservation.

## Author Contributions

MM and SA: data analysis/writing. MM and SD: data collection/writing. RL, ND, CC, and XW: reviewers/editing. All authors contributed to the article and approved the submitted version.

## Conflict of Interest

The authors declare that the research was conducted in the absence of any commercial or financial relationships that could be construed as a potential conflict of interest.

## Publisher's Note

All claims expressed in this article are solely those of the authors and do not necessarily represent those of their affiliated organizations, or those of the publisher, the editors and the reviewers. Any product that may be evaluated in this article, or claim that may be made by its manufacturer, is not guaranteed or endorsed by the publisher.

## References

[1] DollNBorgerMAHainJBuceriusJWaltherTGummertJF. Minimal access aortic valve replacement: effects on morbidity and resource utilization. Ann Thorac Surg. (2002) 74:S1318–22. 10.1016/s0003-4975(02)03911-512400808

[2] ChitwoodWRWixonCLElbeeryJRMoranJFChapmanWHHLustRM. Video-assisted minimally invasive mitral valve surgery. J Thorac Cardiov Sur. (1997) 114:773–80. 10.1016/S0022-5223(97)70081-39375607

[3] Boix-GariboRUzzamanMMBapatVN. Review of minimally invasive aortic valve surgery. Interv Cardiol. (2015) 10:144–48. 10.15420/icr.2015.10.03.14429588692PMC5808565

[4] BouhoutIMorgantMCBouchardD. Minimally invasive heart valve surgery. Can J Cardiol. (2017) 33:1129–37. 10.1016/j.cjca.2017.05.01428843324

[5] MoustafaMAAbdelsamadAAZakariaGOmarahMM. Minimal vs median sternotomy for aortic valve replacement. Asian Cardiovasc Thorac Ann. (2007) 15:472–5. 10.1177/02184923070150060518042770

[6] ArisACamaraMLMontielJDelgadoLJGalanJLitvanH. Ministernotomy versus median sternotomy for aortic valve replacement: a prospective, randomized study. Ann Thorac Surg. (1999) 67:1583–7. 10.1016/s0003-4975(99)00362-810391259

RETRACTED

[7] ChengDCMartinJLalADiegelerAFolliguetTANifongLW. Minimally invasive versus conventional open mitral valve surgery: a meta-analysis and systematic review. Innovations. (2011) 6:84–103. 10.1097/IMI.0b013e3182167feb22437892

[8] MiskovicALumbAB. Postoperative pulmonary complications. Br J Anaesth. (2017) 118:317–34. 10.1093/bja/aex00228186222

[9] WeissmanC. Pulmonary complications after cardiac surgery. Semin Cardiothorac Vasc Anesth. (2004) 8:185–211. 10.1177/10892532040080030315375480

[10] CanetJGallartLGomarCPaluzieGVallesJCastilloJ. Prediction of postoperative pulmonary complications in a population-based surgical cohort. Anesthesiology. (2010) 113:1338–50. 10.1097/ALN.0b013e3181fc6e0a21045639

[11] WeissmanC. Pulmonary function after cardiac and thoracic surgery. Curr Opin Anaesthesiol. (2000) 13:47–51. 10.1097/00000539-199906000-0001417016279

[12] AlbackerTBBlackstoneEHWilliamsSJGillinovAMNaviaJLRoselliEE. Should less-invasive aortic valve replacement be avoided in patients with pulmonary dysfunction?J Thorac Cardiovasc Surg. (2014) 147:355–61. 10.1016/j.jtcvs.2012.12.01423332188

[13] BangJHKimJWLeeJWKimJBJungSHChooSJ. Minimally invasive approaches versus conventional sternotomy for aortic valve replacement: a propensity score matching study. Korean J Thorac Cardiovasc Surg. (2012) 45:80–4. 10.5090/kjtcs.2012.45.2.8022500276PMC3322189

[14] BonacchiMPriftiEGiuntiGFratiGSaniG. Does ministernotomy improve postoperative outcome in aortic valve operation? A prospective randomized study. Ann Thorac Surg. (2002) 73:460–5. 10.1016/s0003-4975(01)03402-611845860

[15] CalderonJRichebePGuibaudJPCoifficABranchardOAsselineauJ. Prospective randomized study of early pulmonary evaluation of patients scheduled for aortic valve surgery performed by ministernotomy or total median sternotomy. J Cardiothorac Vasc Anesth. (2009) 23:795–801. 10.1053/j.jvca.2009.03.01119450991

[16] DoganSAybekTRisteskiPSDethoFRappAWimmer-GreineckerG. Minimally invasive port access versus conventional mitral valve surgery: prospective randomized study. Ann Thorac Surg. (2005) 79:492–8. 10.1016/j.athoracsur.2004.08.06615680822

[17] FarhatFLuZLefevreMMontagnaPMikaeloffPJegadenO. Prospective comparison between total sternotomy and ministernotomy for aortic valve replacement. J Card Surg. (2003) 18:396–401. 10.1046/j.1540-8191.2003.02047.x12974924

[18] GasparovicIArtemiouPHudecVHulmanM. Long-term outcomes following minimal invasive versus conventional aortic valve replacement: a propensity match analysis. Bratisl Lek Listy. (2017) 118:479–84. 10.4149/BLL_2017_09229050486

RETRACTED

[19] GhantaRKLaparDJKernJAKronILSpeirAMFonnerE. Minimally invasive aortic valve replacement provides equivalent outcomes at reduced cost compared with conventional aortic valve replacement: A real-world multi-institutional analysis. J Thorac Cardiovasc Surg. (2015) 149:1060–5. 10.1016/j.jtcvs.2015.01.01425680751PMC4409485

[20] GilmanovDBevilacquaSMurziMCerilloAGGasbarriTKallushiE. Minimally invasive and conventional aortic valve replacement: a propensity score analysis. Ann Thorac Surg. (2013) 96:837–43. 10.1016/j.athoracsur.2013.04.10223866805

[21] GilmanovDFarnetiPAFerrariniMSantarelliFMurziMMiceliA. Full sternotomy versus right anterior minithoracotomy for isolated aortic valve replacement in octogenarians: a propensity-matched study dagger. Interact Cardiovasc Thorac Surg. (2015) 20:732–41. 10.1093/icvts/ivv03025757476

[22] HawkinsRBMehaffeyJHKesselSMDahlJJKronILKernJA. Minimally invasive mitral valve surgery is associated with excellent resource utilization, cost, and outcomes. J Thorac Cardiovasc Surg. (2018) 156:611–16. 10.1016/j.jtcvs.2018.03.10829709359PMC6100741

[23] HiraokaATotsugawaTKuinoseMNakajimaKChikazawaGTamuraK. Propensity score-matched analysis of minimally invasive aortic valve replacement. Circ J. (2014) 78:2876–81. 10.1253/circj.CJ-14-086125421231

[24] HolzheyDMShiWBorgerMASeeburgerJGarbadeJPfannmullerB. Minimally invasive versus sternotomy approach for mitral valve surgery in patients greater than 70 years old: a propensity-matched comparison. Ann Thorac Surg. (2011) 91:401–5. 10.1016/j.athoracsur.2010.08.00621256279

[25] IribarneARussoMJEasterwoodRHongKNYangJCheemaFH. Minimally invasive versus sternotomy approach for mitral valve surgery: a propensity analysis. Ann Thorac Surg. (2010) 90:1471–7. 10.1016/j.athoracsur.2010.06.03420971243PMC9175644

[26] JohnstonDRAtikFARajeswaranJBlackstoneEHNowickiERSabikJF. Outcomes of less invasive J-incision approach to aortic valve surgery. J Thorac Cardiovasc Surg. (2012) 144:852–58. 10.1016/j.jtcvs.2011.12.00822244556

[27] LevackMMAftabMRoselliEEJohnstonDRSolteszEGGillinovAM. Outcomes of a less-invasive approach for proximal aortic operations. Ann Thorac Surg. (2017) 103:533–40. 10.1016/j.athoracsur.2016.06.00827788942

[28] MachlerHEBergmannPAnelli-MontiMDacarDRehakPKnezI. Minimally invasive versus conventional aortic valve operations: a prospective study in 120 patients. Ann Thorac Surg. (1999) 67:1001–5. 10.1016/s0003-4975(99)00072-710320242

[29] MasielloPCoscioniEPanzaATriumbariFPreziosiGDi BenedettoG. Surgical results of aortic valve replacement via partial upper sternotomy: comparison with median sternotomy. Cardiovasc Surg. (2002) 10:333–8. 10.1016/s0967-2109(02)00026-112359403

RETRACTED

[30] MerkDRLehmannSHolzheyDMDohmenPCandolfiPMisfeldM. Minimal invasive aortic valve replacement surgery is associated with improved survival: a propensity-matched comparison. Eur J Cardiothorac Surg. (2015) 47:11–7. 10.1093/ejcts/ezu06824599160

[31] MurziMCerilloAGBevilacquaSGilmanovDFarnetiPGlauberM. Traversing the learning curve in minimally invasive heart valve surgery: a cumulative analysis of an individual surgeon's experience with a right minithoracotomy approach for aortic valve replacement. Eur J Cardiothorac Surg. (2012) 41:1242–6. 10.1093/ejcts/ezr23022232493

[32] SansoneFPuntaGParisiFDatoGMZingarelliEFloccoR. Right minithoracotomy versus full sternotomy for the aortic valve replacement: preliminary results. Heart Lung Circ. (2012) 21:169–73. 10.1016/j.hlc.2011.10.00422071201

[33] SeitzMGoldblattJPaulEMarcusTLarobinaMYapCH. Minimally invasive aortic valve replacement via right anterior mini-thoracotomy: propensity matched initial experience. Heart Lung Circ. (2019) 28:320–26. 10.1016/j.hlc.2017.11.01229291961

[34] ShehadaSEOzturkOWottkeMLangeR. Propensity score analysis of outcomes following minimal access versus conventional aortic valve replacement. Eur J Cardiothorac Surg. (2016) 49:464–9. 10.1093/ejcts/ezv06125732967

[35] StolinskiJMusialRPlicnerDFijorekKMedrzyckiMAndresJ. Respiratory functional status after conventional and minimally invasive aortic valve replacement surgery - a propensity score analysis. Kardiochir Torakochirurgia Pol. (2017) 14:5–9. 10.5114/kitp.2017.6692228515741PMC5404120

[36] StolinskiJPlicnerDGrudzienGWasowiczMMusialRAndresJ. A comparison of minimally invasive and standard aortic valve replacement. J Thorac Cardiovasc Surg. (2016) 152:1030–9. 10.1016/j.jtcvs.2016.06.01227449562

[37] TabataMUmakanthanRCohnLHBolmanRM3rdShekarPSChenFY. Early and late outcomes of 1000 minimally invasive aortic valve operations. Eur J Cardiothorac Surg. (2008) 33:537–41. 10.1016/j.ejcts.2007.12.03718255305

[38] WangQXiWGaoYShenHMinJYangJ. Short-term outcomes of minimally invasive mitral valve repair: a propensity-matched comparison. Interact Cardiovasc Thorac Surg. (2018) 26:805–12. 10.1093/icvts/ivx40229304201

[39] ZhaoDWeiLZhuSJZhangZLiuHYangY. Combined mitral and aortic valve procedure via right mini-thoracotomy versus full median sternotomy insights from a single-center study of propensity-matched data. Int Heart J. (2019) 60:336–44. 10.1536/ihj.18-18630799378

[40] HigginsJPTAltmanDG. Assessing risk of bias in included studies. In: HigginsJPTGreenS, editors. Cochrane Handbook for Systematic Reviews of Interventions. Chichester: Wiley (2008). p. 187–241.

RETRACTED

[41] Ottawa Hospital Research Institu. The Newcastle-Ottawa Scale (nos) for Assessing the Quality of Nonrandomised Studies in Meta-Analyses. (2019). Available online at: http://www.ohri.ca/programs/clinical_epidemiology/oxford.asp (accessed August 14, 2019).

[42] JadadARCarrollDGlynnCJMooreRAMcQuayHJ. Morphine responsiveness of chronic pain: double-blind randomised crossover study with patient-controlled analgesia. Lancet. (1992) 339:1367–71. 10.1016/0140-6736(92)91194-d1350803

[43] GallartLCanetJ. Post-operative pulmonary complications: understanding definitions and risk assessment. Best Pract Res Clin Anaesthesiol. (2015) 29:315–30. 10.1016/j.bpa.2015.10.00426643097

[44] SzelkowskiLAPuriNKSinghRMassimianoPS. Current trends in preoperative, intraoperative, and postoperative care of the adult cardiac surgery patient. Curr Problems Surg. (2014) 52:531–69. 10.1067/j.cpsurg.2014.10.00125524515

[45] TannerTGColvinMO. Pulmonary complications of cardiac surgery. Lung. (2020) 198:889–96. 10.1007/s00408-020-00405-733175990PMC7655908

[46] MoherDLiberatiATetzlaffJAltmanDGGroupP. Preferred reporting items for systematic reviews and meta-analyses: the PRISMA statement. PLoS Med. (2009) 6:e1000097. 10.1371/journal.pmed.100009719621072PMC2707599

[47] CosgroveDM3rdSabikJF. Minimally invasive approach for aortic valve operations. Ann Thorac Surg. (1996) 62:596–7.8694642

[48] BadenesRLozanoABeldaFJ. Postoperative pulmonary dysfunction and mechanical ventilation in cardiac surgery. Crit Care Res Pract. (2015) 2015:420513. 10.1155/2015/42051325705516PMC4332756

[49] ChettaABobbioAAielloMDel DonnoMCastagnaroAComelA. Changes in lung function and respiratory muscle strength after sternotomy vs. laparotomy in patients without ventilatory limitation. Eur Surg Res. (2006) 38:489–93. 10.1159/00009600817008793

[50] e SilvaAMSaadRStirbulovRRivettiLA. Off-pump versus on-pump coronary artery revascularization: effects on pulmonary function. Interact Cardiovasc Thorac Surg. (2010) 11:42–5. 10.1510/icvts.2009.22961720403972

[51] RagnarsdottirMKristjAnsdottirAIngvarsdottirIHannessonPTorfasonBCahalinL. Short-term changes in pulmonary function and respiratory movements after cardiac surgery via median sternotomy. Scand Cardiovasc J. (2004) 38:46–52. 10.1080/1401743031001665815204247

[52] ShenkmanZShirYWeissYGBleibergBGrossD. The effects of cardiac surgery on early and late pulmonary functions. Acta Anaesthesiol Scand. (1997) 41:1193–9.936694310.1111/j.1399-6576.1997.tb04865.x

[53] KhoshbinEPrayagaSKinsellaJSutherlandFW. Mini-sternotomy for aortic valve replacement reduces the length of stay in the cardiac intensive care unit: meta-analysis of randomised controlled trials. BMJ Open. (2011) 1:e000266. 10.1136/bmjopen-2011-00026622116090PMC3225590

RETRACTED

[54] LimJYDeoSVAltarabshehSEJungSHErwinPJMarkowitzAH. Conventional versus minimally invasive aortic valve replacement: pooled analysis of propensity-matched data. J Card Surg. (2015) 30:125–34. 10.1111/jocs.1249325533177

[55] PaparellaDMalvindiPGSantarpinoGMoscarelliMGuidaPFattouchK. Full sternotomy and minimal access approaches for surgical aortic valve replacement: a multicentre propensity-matched study. Eur J Cardiothorac Surg. (2020) 57:709–16. 10.1093/ejcts/ezz28631647535

[56] SantanaOReynaJBenjoAMLamasGALamelasJ. Outcomes of minimally invasive valve surgery in patients with chronic obstructive pulmonary disease. Eur J Cardiothorac Surg. (2012) 42:648–52. 10.1093/ejcts/ezs09822555309

